The article "Overexpression of Wnt7a enhances radiosensitivity of non-small-cell lung cancer via the Wnt/JNK pathway" was retracted in 2022. Reasons: duplicated images; original data or images not available; unreliable data.

# Overexpression of Wnt7a enhances radiosensitivity of non-small-cell lung cancer via the Wnt/JNK pathway

**DOI:** 10.1242/bio.050575

**Published:** 2020-07-01

**Authors:** Pingping Ai, Xianhua Xu, Shijie Xu, Zhixia Wei, Shun Tan, Junzhe Li

**Affiliations:** 1 Department of Pathology, Central South University Xiangya School of Medicine, Affiliated Haikou Hospital, Haikou 570208, Hainan, China; 2 Department of Pathology, Hainan Cancer Hospital, Affiliated Cancer Hospital of Hainan Medical University, Haikou 570311, Hainan, China; 3 Medical Research Center, Hainan Cancer Hospital, Haikou 570311, Hainan, China; 4 Biomedical Research Institute, Seoul National University Hospital, Seoul 03080, Republic of Korea; 5 Department of Oncology, Hainan Cancer Hospital, Affiliated Cancer Hospital of Hainan Medical University, Haikou 570311, Hainan, China; 6 Department of Thoracic Surgery, Hainan Cancer Hospital, Affiliated Cancer Hospital of Hainan Medical University, Haikou 570311, Hainan, China

**Keywords:** Non-small-cell lung cancer (NSCLC), Wnt7a, Radiosensitivity, Wnt/JNK pathway

## Abstract

The Wingless-type protein 7a (Wnt7a) plays an antiproliferative role in non-small-cell lung cancer (NSCLC). Previous studies have indicated that Wnt7a expression was downregulated in radiation-resistant NSCLC cells. However, little is known about its biological functions and molecular mechanisms in radiosensitivity of NSCLC. Thus, NSCLC cell proliferation and apoptosis in response to Wnt7a overexpression and/or radiation were determined by 3-(4, 5-Dimethylthiazol-2-yl)-2, 5-diphenyl-tertazolium bromide (MTT) assay and flow cytometry, respectively. The activation of the Wnt/cJun N-terminal kinase (JNK) and Wnt/β-catenin signaling pathways were further examined by western blot in NSCLC cell lines H1650 and A549. Wnt7a overexpression combined with radiation-inhibited cell proliferation and induced apoptosis in NSCLC cell lines compared to Wnt7a overexpression or radiotherapy alone. In addition, the phosphorylation of JNK, but not β-catenin, was congruent with the changes in Wnt7a overexpression and/or radiation. Moreover, the Wnt/JNK pathway could induce the apoptosis of NSCLC cells through the mitochondrial pathway. Inhibition of the Wnt/JNK signaling pathway by SP600125, a JNK inhibitor, contributed to proliferation induction in NSCLC cells. Taken together, these results showed that Wnt7a overexpression sensitized NSCLC cell lines to radiotherapy through the Wnt/JNK signaling pathway.

## Abstract (precis)

**Summary:** The radiosensitizing effect of Wnt7a in non-small-cell lung cancer (NSCLC).

## INTRODUCTION

Lung cancer is the leading cause of cancer mortality in the world, with non-small-cell lung cancer (NSCLC) accounting for up to 80% of total pulmonary malignancies (Jemal et al., 2011). Radiotherapy is the commonly used treatment for localized lung cancer, and it has the advantage of being non-invasive and well tolerated (Harris et al., 2014; Kim et al., 2017). Radiotherapy plays a crucial role for the local treatment of NSCLC patients including DNA damage, triggering cell cycle arrest, and apoptosis (Palayoor et al., 1995; Ning and Knox, 1999). However, radio-resistance is one major obstacle in the success of radiation treatment. Hence, novel therapeutic strategies to improve the effectiveness of radiation treatment on NSCLC are urgently needed.

The article "Overexpression of Wnt7a enhances radiosensitivity of non-small-cell lung cancer via the Wnt/JNK pathway" was retracted in 2022. Reasons: duplicated images; original data or images not available; unreliable data.

We previously found that the wingless-type (Wnt) pathway was associated with the radio-resistant cells in NSCLC. In particular, Wnt7a expression was most frequently lost in radio-resistant NSCLC cells (Ahn et al., 2014). Wnt7a is a known tumor suppressor gene and is downregulated in NSCLC cells (Yoshioka et al., 2012; Winn et al., 2006). In addition, restoration of Wnt7a expression inhibits the proliferation of NSCLC cells (Winn et al., 2005). Thus, the main purpose of the present study is to evaluate the efficacy of Wnt7a overexpression combined with radiotherapy in NSCLC cell lines, because preclinical and clinical studies have reported that the combination of gene therapy and conventional anticancer therapy can improve therapeutic benefit (Fang and Roth, 2003).

Previous research suggests that Wnt/β-catenin pathway may modulate the radiosensitivity of NSCLC cells. For example, knockdown of Thyroid cancer 1 sensitizes NSCLC cell lines to radiotherapy through the Wnt/β-catenin signaling pathway (Wu et al., 2016). In addition, GDK-10017, an inhibitor of the Wnt/β-catenin signaling pathway, causes significant radiosensitivity of NSCLC cells (Wickham et al., 1997). Moreover, loss of Wnt transcription factor TCF4 enhances sensitization of cancer cells to radiotherapy (Jacob et al., 2004). However, a previous study demonstrated that overexpression of Wnt7a inhibited NSCLC cell proliferation through the cJun N-terminal kinase (JNK) pathway but not the β-catenin pathway (Winn et al., 2005). The JNK pathway can be induce by various stimuli, such as UV irradiation, cytokine, oxidative stress and chemotherapeutic drugs (Davis, 2000; Karin, 1998; Hagemann and Blank, 2001). Therefore, the activities of β-catenin and JNK pathways were also examined to elucidate whether re-expression of Wnt7a leads to sensitization to radiotherapy for NSCLC via the Wnt/β-catenin or Wnt/JNK pathways.

## RESULTS

### Wnt7a overexpression enhanced the inhibition of NSCLC cell proliferation to irradiation

To investigate the effects of Wnt7a overexpression on radiation-induced anti-tumor therapy in NSCLC cell lines H1650 and A549, the MTT assay was used to determine the proliferation of cells transfected with pcDNA6-Wnt7a or empty vector control combined with radiation or radiation alone. Wnt7a induced the cellular transformation through its receptor Fzd-9 (Tennis et al., 2012; Winn et al., 2005), we thus examined the expressions of Wnt7a and Fzd-9 to select stable expression clones. Immunoblot and RT-PCR were used to confirm Wnt7a and Fzd-9 expressions (Fig. 1A). Treatment with ionizing radiation (IR, 2–8 Gy) alone inhibited the dose-dependent changes in H1650 and A549 cell growth (Fig. 1B). Moreover, overexpression of Wnt7a (60.2% in H1650, 59.8% in A549) displayed lower proliferation rates compared with cells with empty vector control (23.9% in H1650, 21.8% in A549), and empty vector control had no significant effect on the cell proliferation compared with radiation alone. Thus, these data indicated that a combination of Wnt7a overexpression and irradiation improved the cell-killing effect of NSCLC cell lines.

The article "Overexpression of Wnt7a enhances radiosensitivity of non-small-cell lung cancer via the Wnt/JNK pathway" was retracted in 2022. Reasons: duplicated images; original data or images not available; unreliable data.

**Fig. 1.** **Wnt7a overexpression sensitized H1650 and A549 cells proliferation to irradiation.** (A) Stable expression of Wnt7a in transfected H1650 and A549 cells were verified by RT-PCR and by immunoblot with the Fzd-9 and GAPDH loading control. Data are expressed as the fold change of control cells (empty vector) and normalized to the corresponding GAPDH level. (B) Proliferation rate calculated for H1650 and A549 cell lines. The cell proliferation rate was determined by the MTT assay after irradiation. The data shown are the average of triplicate experiments.

### Wnt7a overexpression induced the apoptosis by irradiation in NSCLC cell lines

To determine whether Wnt7a overexpression sensitized the apoptosis of H1650 and A549 cells to irradiation, cells were transfected with pcDNA6-Wnt7a and then irradiated with either 0 or 4 Gy. After 24 h, the percentage of apoptotic cells was determined by Annexin V/Propidium Iodide apoptosis analysis (Fig. 2). Apoptosis rates in H1650 and A549 cell with Wnt7a overexpression (6.74% in H1650, 4.66% in A549) or irradiation (2.74% in H1650, 8.50% in A549) alone were significantly increased compared with control cells (*P*<0.05). In addition, a combination of Wnt7a overexpression and irradiation (19.74% in H1650, 25.67% in A549) resulted in an enhanced increase in the induction of apoptosis. This data demonstrated that Wnt7a overexpression sensitized the apoptosis of NSCLC cell lines to irradiation.

**Fig. 2.** **Wnt7a overexpression sensitized H1650 and A549 cell apoptosis to irradiation.** Apoptosis was detected by Annexin V staining in the H1650 (A) and A549 (B) NSCLC cell lines. Apoptosis rates were significantly higher in the combination with Wnt7a overexpression and irradiation than other groups. ^a^*P*<0.05 compared to control group, ^b^*P*<0.05 compared to irradiation group, ^c^*P*<0.05 compared to Wnt7a overexpression group.

The article "Overexpression of Wnt7a enhances radiosensitivity of non-small-cell lung cancer via the Wnt/JNK pathway" was retracted in 2022. Reasons: duplicated images; original data or images not available; unreliable data.

### Combination of Wnt7a overexpression and irradiation activated the JNK pathway but not the β-catenin pathway in NSCLC cell lines

To test whether Wnt7a overexpression and irradiation inhibited the proliferation and induced the apoptosis in NSCLC cells through the JNK or β-catenin pathways, we examined the phosphorylation levels of JNK (Thr183/Tyr185) and β-catenin (Thr-41/Ser-45, Ser-552, Ser-675 and Ser-45) by western blot (Fig. 3). We revealed that the phosphorylation level of JNK (Thr183/Tyr185) was elevated by Wnt7a overexpression or irradiation alone in H1650 and A549 cells compared with control group (*P*<0.05). Additionally, a combination of Wnt7a overexpression and irradiation further enhanced the already increased phosphorylation level of JNK (Thr183/Tyr185). On the other hand, phosphorylation levels of β-catenin (Thr-41/Ser-45, Ser-552, Ser-675 and Ser-45) were only affected by irradiation treatment in H1650 and A549 cells. Thus, these results suggest that a combination of Wnt7a overexpression and irradiation could affect the JNK pathway in NSCLC but not β-catenin activity.

**Fig. 3.** **Effect of Wnt7a overexpression and irradiation on the phosphorylation of JNK, β-catenin in H1650 and A549 NSCLC cell lines.** The expression of p-JNK (Thr183/Try185), JNK (total), β-catenin (Thr41/Ser45), β-catenin (Ser552), β-catenin (Ser675), β-catenin (Ser45) and β-catenin (total) were determined by western blot analysis. Representative immunoblots by transfection with Wnt7a and/or irradiation (4 Gy). The phosphorylation level of JNK was increased with the combination of Wnt7a overexpression and irradiation than with Wnt7a overexpression or irradiation alone. GAPDH was used as a loading control.

### SP600125, a JNK inhibitor, reversed the inhibition of NSCLC cell proliferation by Wnt7a overexpression

To examine the role of the JNK pathway in NSCLC cell growth inhibition induced by Wnt7a overexpression and irradiation, H1650 and A549 cells were treated with 50 µM SP600125. Fig. 4A demonstrated the constitutive treatment with SP600125 in H1650 and A549 cells and that the phosphorylation level of JNK (Thr183/Tyr185) was decreased. H1650 and A549 cells treated with SP600125 blocked the reduced proliferation of NSCLC cells by the combination of Wnt7a overexpression and irradiation (Fig. 4B). Therefore, this data indicated that the JNK pathway is a likely mediator of the decreased proliferation stimulated by Wnt7a overexpression and irradiation.

The article "Overexpression of Wnt7a enhances radiosensitivity of non-small-cell lung cancer via the Wnt/JNK pathway" was retracted in 2022. Reasons: duplicated images; original data or images not available; unreliable data.

**Fig. 4.** **Inactivation of the Wnt/JNK signaling pathway reversed the inhibition of cell proliferation by the combination of Wnt7a overexpression and irradiation.** (A) The expression of p-JNK (Thr183/Try185) and JNK (Total) were determined by western blot analysis in H1650 and A549 cells treated with SP600125. (B) Proliferation rate calculated for H1650 and A549 treated with SP600125 and/or Wnt7a overexpression. The cell proliferation rate was determined by the MTT assay after irradiation (4 Gy). Results are representative of triplicate experiments.

### Wnt7a overexpression sensitized the irradiation for NSCLC via the mitochondrial pathway of apoptosis

To further elucidate whether Wnt7a overexpression sensitized irradiation was associated with the mitochondria-dependent apoptotic pathway in NSCLC cell lines, we examined the expression of caspase-3, caspase-7, caspase-9, PARP, Bcl-2, Bax and cytochrome *c* induced by the combination of Wnt7a overexpression and irradiation (Fig. 5). The expression levels of caspase-3, caspase-7, caspase-9, PARP, Bax and cytochrome *c* were prominent in the combination of Wnt7a overexpression and irradiation relative to Wn7a overexpression or irradiation alone. On the contrary, expression of Bcl-2 was suppressed in the combination of Wnt7a overexpression and irradiation relative to Wn7a overexpression or irradiation alone. Thus, these results indicated that a combination of Wnt7a overexpression and irradiation enhanced the apoptosis of NSCLC cells via the mitochondrial pathway.

**Fig. 5.** **The combination of Wnt7a overexpression and irradiation induced the apoptosis in H1650 and A549 NSCLC cell lines through the mitochondrial pathway.** The expression of PARP, caspase-3, caspase-7, caspase-9, Bcl-2, Bax and cytochrome *c* were determined by western blot analysis. Representative immunoblots by transfection with Wnt7a and/or irradiation (4 Gy). The expression of PARP, caspase-3, caspase-7, caspase-9, Bax and cytochrome *c* were more prominent with the combination of Wnt7a and irradiation than with Wnt7a overexpression or irradiation alone. The expression of Bcl-2 was suppressed with the combination of Wnt7a and irradiation than with Wnt7a overexpression or irradiation alone. GAPDH was used as a loading control.

## DISCUSSION

Previous studies have reported that Wnt7a expression was downregulated in NSCLC cells (Ahn et al., 2014), which indicated the tumor-protective role of Wnt7a in biological functions (Bikkavilli et al., 2015; Winn et al., 2005). A previous study demonstrated that re-expression of Wnt7a reduced the proliferation of NSCLC cells (Winn et al., 2005). Thus, we hypothesized that overexpression of Wnt7a might sensitize NSCLC cell lines to radiation therapy. To confirm this hypothesis, we overexpressed Wnt7a by transfecting Wnt7a-pcDNA6 in NSCLC cell lines H1650 and A549. Our data showed that Wnt7a overexpression combined with irradiation inhibited cell proliferation and induced apoptosis in NSCLC cell lines more than the irradiation alone (Figs 1 and 2). Therefore, these results suggest that the combination of Wnt7a overexpression and radiotherapy has a synergistic effect on therapeutic strategies for NSCLC.

The article "Overexpression of Wnt7a enhances radiosensitivity of non-small-cell lung cancer via the Wnt/JNK pathway" was retracted in 2022. Reasons: duplicated images; original data or images not available; unreliable data.

We demonstrated that Wnt7a overexpression in combination with irradiation inhibited cell proliferation and induced apoptosis in NSCLC cells through activation of the JNK pathway but not the β-catenin signaling pathway. Our results showed that Wnt7a failed to engage the β-catenin pathway, which is consistent with a previous study demonstrating that Wnt7a stimulates the JNK pathway but not β-catenin activity in NSCLC cells (Winn et al., 2005). In addition, we found that JNK inhibitor SP600125 reduced the proliferation of NSCLC cells by the combination of Wnt7a overexpression and irradiation. JNKs are widely invoked as components of pro-apoptotic signaling cascades (Kennedy et al., 2003), and the JNK pathway promotes an epithelial cell differentiation program in lung cancer cells (Xia and Karin, 2004). It is well known that the activation of JNK pathway by UV irradiation induces apoptosis (Karin, 1998). Thus, these results suggest that the Wnt/JNK pathway plays a critical role in radiotherapy sensitization of NSCLC.

The apoptosis pathway can be divided into two major pathways: the intrinsic and extrinsic pathways (Elmore, 2007). The intrinsic pathway is activated by various cellular stresses such as radiation exposure and growth factor withdrawal (Green and Llambi, 2015). The intrinsic pathway is mitochondria-mediated apoptosis that initiates apoptosis signaling by binding to the Bcl-2-like pro-survival proteins (including Bcl-2 and Bcl-xL) and releases Bax to promote the loss of mitochondrial outer membrane potential, cytochrome *c* release and activation of caspase-9 and caspase-3, resulting in apoptosis (Oltval et al., 1993; Lotem and Sachs, 1993; Karna et al., 2009; Hotchkiss et al., 2009; Strasser, 2005). Our results indicated that the combination of Wnt7a overexpression and irradiation decreased the Bcl-2 expression, increased the activation of Bax, caused the release of cytochrome *c*, and enhanced the activation of caspase-3, caspase-7 and caspase-9 in NSCLC cells (Fig. 5). Thus, these results indicate that Wnt7a overexpression enhances apoptosis-inducing effects of radiotherapy on NSLCL cells via the activation of the mitochondrial pathway of apoptosis.

The article "Overexpression of Wnt7a enhances radiosensitivity of non-small-cell lung cancer via the Wnt/JNK pathway" was retracted in 2022. Reasons: duplicated images; original data or images not available; unreliable data.

## CONCLUSION

In conclusion, the results of the present study suggest that Wnt7a overexpression in combination with irradiation enhanced the inhibition of cell proliferation and induction of apoptosis in NSCLC cells via the Wnt/JNK signaling pathway, thereby improving the susceptibility of NSCLC to radiotherapy. The radiosensitizing effect of Wnt7a overexpression induces apoptosis of NSCLC that is mitochondrially-driven and is executed through the activated caspase by the cleavage of downstream targets. The combination of Wnt7a gene therapy and irradiation may be a feasible and effective radiosensitizer for the treatment of NSCLC.

## MATERIALS AND METHODS

### Cell culture

Human NSCLC cell lines H1650 (ATCC CRL-5883) and A549 (ATCC CCL-185) were purchased from American Type Culture Collection (ATCC; Manassas, VA, USA). The cells were cultured in RPMI-1640 (Life Technologies, Carlsbad, CA, USA) containing 10% fetal calf serum and 1% penicillin/streptomycin in culture dishes at 37°C in a humidified atmosphere with 5% CO_2_. Cells (5×10^5^/well) were seeded on to six-well culture plates.

### Overexpression of Wnt7a in lung cancer cell lines

pcDNA6-Wnt7a plasmid was constructed by subcloning the fragment of the Wnt7a-encoding cDNA from plasmid pOTB7-Wnt7a (KRIBB. Daejeon, Korea) into pcDNA6 at the *Kpn* I and *Xba* I sites. For the transfection, approximately 1.0×10^5^ A549 and H1650 parental cells were seeded in six-well plates. When the cells reached 80–90% confluence, the cells were transfected with pcDNA6-Wnt7a and pcDNA6-empty using EzWay™ Transfection Reagent (Komabiotech, Korea), according to the manufacturer's instructions. The ratio of the plasmids to the transfection reagent was 1 μg:3 μl. At 48 h post-transfection, 20 μg/ml Blasticidin (Sigma-Aldrich, St Louis, MO, USA) was added to select stable transfections.

### Radiation treatment and reagent

48 h post-transfection, cells were irradiated (0, 2, 4, 6 or 8 Gy in a single fraction) with 6 MV photon beams produced by a 21 EX (Varian, Palo Alto, CA, USA) linear accelerator. Cells were then cultured for a further 24 h before being examined by flow cytometry and western blot analysis. The specific inhibitor of JNK (SP600125, Selleck Chemicals, Houston, TX, USA) was dissolved in DMSO.

### Cell proliferation assay

The cell proliferation assay was measured by 3-(4, 5-Dimethylthiazol-2-yl)-2, 5-diphenyl-tertazolium bromide (MTT) assay. 48 h post-transfection, cells were treated with irradiation, then cultured in 6-well culture plates and incubated for 5 days under standard conditions (37°C in a humidified atmosphere containing 5% CO_2_). After 5 days, an aliquot of 10 μl MTT (5 mg/ml in phosphate-buffered saline, Sigma-Aldrich) was added to each well. After 2 h of incubation at 37°C, 100 μl/well isopropanol with 40 mM HCl was added. Optical density was read at 560 nm and 620 nm on a measurement parameter editor (Tecan, Grodig, Austria).

The article "Overexpression of Wnt7a enhances radiosensitivity of non-small-cell lung cancer via the Wnt/JNK pathway" was retracted in 2022. Reasons: duplicated images; original data or images not available; unreliable data.

### Cell apoptosis assay

Cell apoptosis was determined by Annexin V-FITC and PI stain. 24 h after treatment with irradiation, cells were re-suspended in 100 μl binding buffer [10 mM HEPES (N-2-hydroxyethylpiperazine-N-2-ethanesulfonic acid), 140 mM NaCl and 2.5 mM CaCl_2_, pH 7.4]. Cells were then stained with 5 μl Annexin V-FITC (BD, Franklin Lakes, NJ, USA) and 5 μl propidium iodide (BD) staining solution in the dark at room temperature for 15 min. The cell samples were analyzed by flow cytometry (Beckman Coulter, CA, USA).

### Western blot analysis

Cells were harvested and protein was extracted using lysis buffer (M-PER Mammalian Protein Extraction Reagent; Thermo Fisher Scientific, Rockford, IL, USA). The Bradford method (Bio-Rad Laboratories, Hercules, CA, USA) was used for protein quantification. Equal amounts of protein were separated by SDS-polyacrylamide gel electrophoresis and transferred to a polyvinylidene difluoride (PVDF) membrane (GE Healthcare, Little Chalfont, UK). The membrane was blocked with blocking buffer containing 5% skim milk in TBS-T (0.1% Tween 20 in TBS) for 1 h at room temperature and then incubated with primary antibodies overnight at 4°C. The membranes were then incubated with secondary antibodies for 1 h at room temperature. Primary antibodies against PARP, caspase-3, caspase-7, caspase-9, Bcl-2, p-Thr-41/Ser-45-β-catenin, p-Ser-552-β-catenin, p-Ser-675-β-catenin, p-Ser-45-β-catenin, β-catenin, p-Thr-183/Thy-185-JNK, JNK, Bax, cytochrome *c* (Cell Signaling Technology; Danvers, MA, USA), Frizzled-9 (Fzd-9; Abcam, Cambridge, MA, USA) and GAPDH (Santa Cruz Biotechnology; Santa Cruz, CA, USA) were used to dilutions of 1:800 to 1:2000. Anti-rabbit or mouse IgG was used as the secondary antibody (Jackson ImmunoResearch, West Grove, PA, USA). Reactive bands were detected by chemiluminescence kit (EMD Mililpore, Billerica, MA, USA). Immunoreactive bands were visualized on membranes by using the Las-4000 system (Fujifilm, Tokyo, Japan).

### Reverse transcription-PCR analysis of Wnt7a mRNA expression

Total cellular RNA was isolated using Trizol reagent according to the manufacturer's protocol (Invitrogen, Carlsbad, CA, USA). RT-PCR was performed with total RNA (2 mg) using the First Strand RT-PCR Kit (Promega, Fitchburg, WI, USA). cDNA was amplified by PCR using specific primers for the target genes, and glyceraldehyde 3-phosphate dehydrogenase (GAPDH) was also amplified as an internal standard. The thermal cycles were as follows: 1 cycle at 95°C for 3 min, 30 cycles at 95°C for 40 s, 58°C for 40 s and 72°C for 90 s, followed by a final elongation step at 72°C for 10 min. The corresponding primer sequences were as follows: Wnt7a, 5′-ATGCCCGGACTCTCATGAAC-3′ and 5′-GTCTTGGTGGTGCACGAGC-3′; Fzd-9, 5′-GCAGTAGTTTCCTCCTGACCG-3′ and 5′-TCTCTGTGTTGGTGCCGCC-3′; GAPDH, 5′-ACCACAGTCCATGCCATCAC-3′ and 5′-TCCACCACCCTGTTGCTGTA-3′. RT-PCR products were electrophoresed through a 1.5% agarose gel with ethidium bromide. Signals were quantified by densitometric analysis using the Labworks Image Acquisition (UVP, Upland, CA, USA). Quantification of Wnt7a gene expression was based on densitometry readings. Statistical analysis was performed to calculate the gel intensity using Microsoft Excel software (Microsoft, Redmond, WA, USA).

The article "Overexpression of Wnt7a enhances radiosensitivity of non-small-cell lung cancer via the Wnt/JNK pathway" was retracted in 2022. Reasons: duplicated images; original data or images not available; unreliable data.

### Statistical analysis

All data were derived from at least three independent experiments. The data were expressed as means±standard deviation (s.d.). Statistical analyses were performed using One-way analysis of variance (ANOVA) or Student's *t*-test. All analyses were performed using the version 21.0 SPSS software package for Windows (SPSS Inc.; Chicago, Illinois, USA), and *P*-values <0.05 were considered to be statistically significant.
